The article "Understanding the Impact of Transformational Leadership on Project Success: A Meta-Analysis Perspective" was published in 2021. Journal: Comput Intell Neurosci.

# Understanding the Impact of Transformational Leadership on Project Success: A Meta-Analysis Perspective

**DOI:** 10.1155/2021/7517791

**Published:** 2021-10-18

**Authors:** Na Zhao, Dongjiao Fan, Yun Chen

**Affiliations:** ^1^School of Traffic and Transportation Engineering, Changsha University of Science and Technology, Changsha 410114, China; ^2^Engineering Research Center of Catastrophic Prophylaxis and Treatment of Road and Traffic Safety of Ministry of Education, Changsha University of Science and Technology, Changsha 410114, China

## Abstract

This paper aims to systematically analyze the reasons for the differences in the relationship between transformational leadership (TL) and project success and apply meta-analysis to summarize which dimensions of TL are the main driving forces for project success. Adopting the meta-analysis approach, we investigated 31 independent studies (*N* = 6475) and studied the theoretical moderators of this relationship from the perspectives of mediating variables, cultural background, and document type to test whether the moderating effects can explain the inconsistent research results. The results reveal that TL positively affects project success and leadership charm is the primary driver of TL. Also, the existence of a mediating mechanism has a more significant impact on the success of the leading project. Meanwhile, compared with project construction under the Western cultural background, countries with Eastern culture are more inclined to use a people-oriented philosophy for project management to promote project success. This research provides an empirical perspective to help project leaders select management talents, regulate leaders' words and deeds, and cultivate technical and soft leadership skills. Besides, this paper proposes a unique and nuanced view of the relationship between TL and project success, enhancing people's understanding of the TL's role in influencing project success.

## 1. Introduction

“Construction Industry 4.0,” as a part of “Industry 4.0,” is a specific application under the subdivision of the construction industry. It mainly contains two themes: “smart factory” and “smart production.” With the emergence of the intelligent construction concept, a plenty of new-generation information technologies, such as 5G, construction robots, and BIM, have been applied in construction projects [1–3]. The integration of technologies has led to a gradual shift in project management from mechanization and digitalization to informatization and intelligence. However, many studies have shown that even with the increasing level of technology and management associated with project construction, the level of project success has not improved significantly due to the increasing complexity and uncertainty of the construction environment. For construction companies and project organizations, changes in production models require far-reaching strategic decisions at all levels of the construction industry. Therefore, it is necessary to change the project organization to achieve a higher level of sustainable project success. It is well known that leaders play a dominant role in project organization reform, which is essential to increase organizational resilience and agility and develop high-reliability organizations [4]. Particularly in the last decade, an increasing number of project operations have developed under the project manager responsibility system. The project manager undertakes the leadership responsibility for the entire process of project implementation and overall management. This change will inevitably affect the leadership behavior of project managers and put forward higher requirements for their ability and comprehensive quality. Compared with other leadership styles, transformational leadership (TL) has advantages in enhancing project success. For example, it attaches great importance to the leaders' standards of behavior and concerns for the needs of followers. Meanwhile, many reasons suggest that TL is indispensable in project organizational change [5–7]. Bass [8] argued that today's construction environment requires subordinates to perform beyond ordinary expectations, and TL can deliver. Therefore, both subordinates and superiors of the project believe that leaders with a transformational style are more productive and suitable for project managers [9].

In recent years, many scholars have conducted many empirical studies to explore the role of TL in project success [10, 11]. On the one hand, most researchers have shown that TL can promote project success. Zhang et al. [12] summarized the recent research results of some scholars and believed that TL plays a vital role in project success or failure. Appropriate TL is necessary for individuals or groups to carry out innovative behaviors [13]. Odusami et al. [14] conducted research to suggest a remarkable correlation between project managers' professional level, leadership style, team composition, and project success. Berssaneti et al. [15] pointed out that project success depends on many factors, including leadership ability, leadership style, and leadership skills of the project manager. However, on the other hand, some studies are reckoning that the project's successful realization will be hindered by TL [16–18]. Zhang [19] found an inhibitory relationship between the project manager's emotional intelligence and leadership style. Iqbal et al. [20] conducted surveys and interviews with engineering organizations in Malaysia. They believed that project leaders' high degree of psychological empowerment negatively impacted project performance due to their leadership style. Besides, Chen et al. [21] proposed an inverted U-shaped relationship between TL and project success, which suggests that it is most conducive to improving the project success rate when TL is at a medium level.

According to the discussion above, there are apparent conflicts in the strength, direction, and statistical significance of the relationship in most studies, which creates confusion in theory and practice. The scholars have not yet formed a consistent perspective on the relationship between TL and project success. Furthermore, the existing research lacks a more systematic and comprehensive integration of TL that contributes to project success, as well as fails to analyze and explain the differences in findings. Simultaneously, the impact of different dimensions of TL on the project's success has not yet been explored by scholars from the perspective of meta-analysis. Therefore, this paper intends to adopt a meta-analysis method through the comprehensive reanalysis of different individual research results to examine the overall effect of TL and other dimensions of TL on project success. Based on the literature collation results, this study explores mediating variables, cultural factors, and publication type factors as the moderating variables, focusing on identifying the reasons for the divergence between different research variables. The research conclusions are expected to comprehensively evaluate TL's theoretical and practical value in construction projects and inspire the sustainable development of project management practices in construction enterprises.

The remainder of the paper is structured as follows: Section 2 sums up the theoretical literature.  Section 3 describes the methodology and the process of data collection.  Section 4 analyses the results of the meta-analysis. A detailed discussion, implication, and limitation are provided in Section 5. Finally, Section 6 concludes this paper and points out the future research direction.

## 2. Literature Review and Hypotheses Development

### 2.1. Transformational Leadership

Burns proposed TL in 1978, and then Bass defined and quantified it in 1985 [8]. According to Bass, TL means that the leaders use words and actions to make subordinates realize the meaning and value of their work [22]. In this process, leaders also create a working atmosphere of trust and cooperation to inspire subordinates' enthusiasm for success and self-realization. In this way, the project manager can encourage them to surpass their interests for the organization's benefit to work more and improve their personal and organizational interests as well as the society's common well-being.

At present, most of the research on TL has been influenced by Bass. Although the multidimensionality of the transformational leader structure has been controversial [23, 24], with the gradual intensification of the discussion on TL, experts and scholars have extended the research from qualitative to quantitative and gradually presented different measurement dimensions of TL. Bass [22] initially proposed that the dimensions of TL have charm, intellectual stimulation, and individualized consideration. After that, Bommer [23] developed the integration, high-performance implementation, and personalized support. Also, Bass and Avolio [24] thought it includes charm, charisma, intellectual stimulation, and individualized consideration. Eventually, Li [25] proposed that TL can be divided into four dimensions: idealized influence, intellectual stimulation, leader charism, and individualized consideration, and they are widely accepted and used. Based on the discussion above, TL is embodied in four dimensions in this paper: (1) idealized influence, which draws a future blueprint for team members, and strengthens team beliefs; (2) intellectual stimulation, which clarifies team goals and encourages members to continue to cooperate in their work, practice, and innovation; (3) leadership charisma, which enhances the self-confidence, self-esteem, and autonomy of members; (4) individualized consideration, which can improve employee identification, loyalty, and enthusiasm.

### 2.2. Project Success

Nowadays, project management has become ubiquitous in the construction industry, capacity building, and social projects [26]. Project success was introduced in the research field of project management in the 1960s and was initially applied for project management performance. Many scholars have defined project success with deepening the research, but they have not yet come to a consistent conclusion. This article summarizes the opinions of essential project management scholars and practitioners on the definition of project success based on the published literature (Table 1).

However, as project functions and the number of stakeholders has ascended, project success has a broader concept, which must be a multidimensional structure [34, 35]. Therefore, the Project Management Institute (PMI) defines project success to balance the competing demands for project quality, scope, time, and cost, as well as meet project stakeholders' changing concerns and expectations (PMI, 2008). Specifically, it includes the organization's benefits, user satisfaction, the benefits to project personnel, sustainability, and business success. Specific to the engineering project, the stakeholders have not formed a unified opinion on the project's success. The main reason is that many stakeholders involved in the project have inconsistent standards about project success and an extended project success evaluation period.

At the same time, scholars now no longer only focus on complex indicators such as quality, schedule, and cost for measuring project success but start to explore soft indicators, such as whether the partnership is enhanced, whether the company's capabilities have improved, and whether there is a willingness to cooperate next time, etc.

### 2.3. Transformational Leadership and Project Success

Many scholars, such as Nam [36], Khawaja et al. [37], and Wang et al. [38], have supported leadership as a critical factor in promoting project success. Empirical evidence generally recognises the positive impact of TL on follower attitudes, effort, and performance. According to Bass and Avolio [39], TL motivates their subordinates to do things that not only exceed what they are simply asked to do, but also the effects often exceed their expectations. Simultaneously, in addition to directly affecting the performance of cross-level followers, TL can also indirectly affect project performance through direct subordinate leaders who contact cross-level followers [40]. Singh [41] postulated that the intellectual stimulation dimension of TL enhances exploratory thinking and communicates a clear vision of the project, motivating project members to generate new ideas.

Moreover, the leaders who demonstrate TL can gain their immediate followers [9] and are increasingly confident in trying new methods to complete projects with the support of their managers. Dulaimi [41] found that the leader's charisma and innovation support behavior are the main reasons for the investigated project's success in Singapore. Also, literature reviews show that project managers' individualized care and idealized influence play a vital role in achieving tremendous project success [42, 43]. Therefore, according to the findings above, this research proposes the following hypotheses:

  H1: TL positively affects project success
  H2a: leader charisma positively affects project success
  H2b: idealized influence positively affects project success
  H2c: intellectual stimulation positively affects project success
  H2d: individualized care positively affects project success

### 2.4. Moderating Relationships

Due to independent research's heterogeneity, certain potential control variables may affect the relationship between TL and project success. This paper summarizes the literature in this article and finds that the literature has differences in mediating variables, cultural background, and publication types.

#### 2.4.1. The Existence of Mediating Variables

Many studies have used mediating variables when discussing the relationship between TL and project success. Chou [44] used cognitive trust and collective effectiveness as intermediary variables to reveal the interrelationship between TL and team performance. Furthermore, García-Morales et al. [45] analyzed the impact of TL on organizational performance through organizational learning and innovation's dynamic capabilities. Aga and Vallejo [46] adopted a field survey with a sample of 200 development project managers in Ethiopian nongovernmental organization (NGO) departments. It adopted the structural equation model to find that team building plays a mediating role between TL and project success. Hassan et al. [47] saw that leaders apply their skills and abilities to contribute to the success of construction projects in Pakistan in project management. Thus, based on the existing literature, this study proposed the following hypothesis:

  H3: the existence of mediating variables moderates the relationship between TL and project success

#### 2.4.2. Document Type

As the relationship between TL and project success varies across studies, the meta-analysis literature includes both published journal articles and unpublished papers. Therefore, the type of literature publication may be a source of variation. Furthermore, the earlier the published research, the more likely it will report significant training effects [48]. Meanwhile, the uncertainty and controversy gradually become clear through the in-depth analysis. Compared to unpublished literature such as thesis, the journal papers are more inclined to describe significant results and distort the natural effect to avoid becoming drawer files [49]. Therefore, this paper proposes the following hypothesis:

  H4: the document type moderates the relationship between TL and project success

#### 2.4.3. Cultural Background

Culture is a consciousness system gradually formed by human beings through coping with problems and adapting to the social development. It shapes not only humans' behavior but also influences humans' psychological needs. The leaders' attitudes, behaviors, and motivations towards their subordinates will vary depending on their culture [50].

These cultural differences will also impact the effectiveness of leadership behavior [51]. Western culture is mainly influenced by European and American cultures, which actively encourages people to express their visions and tendencies in organizations and promotes individualism. However, Eastern culture is more affected by Confucian patriarchal culture, and it advocates collectivism more than Western civilization, especially during the construction of large-scale projects [3]. The project teams can collaborate and cooperate based on task interdependence to promote the efficient integration of heterogeneous innovation resources. On the other hand, the samples used in different studies usually come from different countries. The differences in the countries' economic level and cultural environment where the models belong have a particular impact on the project's successful realization [52, 53]. Therefore, the following hypothesis is formulated:

  H5: cultural background moderates the relationship between TL and project success, and TL in developed countries has a more significant impact on project success

According to the above assumptions, this study proposed a theoretical research model, shown in Figure 1.

## 3. Method and Data

In recent years, meta-analysis has contributed prominently to the literature review as a new method of combining empirical research with research hypotheses. Specifically, meta-analysis can reanalyze multiple empirical research results with the same research purpose to obtain the fundamental relationship between variables. The advantage of meta-analysis is that it can systematically analyze many documents and evaluate the inconsistency of different research results [54]. This method can discover and explain the differences between various research results, systematically integrate the existing empirical research results, and further improve its reliability and validity. Therefore, this paper mainly uses Hunter and Schmidt's primary effect test as well as moderating effect test method. It adopts CMA 2.0 software to assist with the version bias heterogeneity test.

### 3.1. Literature Sources and Collection

According to the following three steps, this research points to the literature collection to ensure the systematic literature collection. Firstly, this study shows computerized keyword searches in the databases Web of Science, Google Scholar, Science Direct, Elsevier, and Springer before October 2020. The papers are searched by the following keywords: “transformational leadership,” “project success,” “project manager,” and “Construction project success.” Secondly, to avoid the omission of essential documents since some related studies on TL and project success are not included in the above databases, this research combines the collected records with the references of these documents, especially compared to the review literature one by one. Finally, the study manually searches the most essential and relevant journals, such as “*Journal of Cleaner Production*,” “*The Leadership Quarterly*,” and “*International Journal of Project Management*.”

The process and results are shown in Figure 2.

### 3.2. Literature Inclusion Criteria

The searched documents are filtered according to the following criteria: (1) It must be a survey or experimental empirical research, excluding pure theoretical and literature review articles. (2) It uses both the TL measurement scale and the project success measurement scale, and at least reports the correlation coefficient (*r*) between the dimension or total score of one scale and the dimension or total score of another scale. Or it can be converted into the *F*-value, *t*-value, or *X*^2^ value of *r*. (3) The selected research is not only limited to journal papers, but also includes thesis, book chapters, etc. (4) If the data is published repeatedly, the published journal articles shall be taken. (5) Document effect value encodes an effect value based on each independent sample.

### 3.3. Document Coding Content and Results

The subsamples included in the meta-analysis are also ordered as follows: firstly, the necessary information of the research (author name and publication time), sample size, and whether there are intermediate variables in the empirical research (divided into yes and no), the cultural background of the study (divided into Eastern culture, Western culture, and others) and the type of article (journal papers, thesis).

Secondly, the research should primarily discuss the total effect of TL on project success. This paper adopts the weighted average method for the influence coefficients of different dimensions of TL mentioned in the literature on project success. If they encounter the literature that discusses the disparate dimensions of TL on project success, the final effect value would be obtained by taking the average layer by layer. The necessary coding information of the main effects analysis is shown in Table 2.

## 4. Results

### 4.1. Test for Publication Bias

Funnel plots are the most commonly used approach to determine the presence of publication bias.  Figure 3 shows the distribution of the effect value. It can be seen that most of the samples concentrate at the top of the funnel chart, and the scattered points distribute near the effect value [55]. Therefore, the possibility of publication bias in this study is relatively slight. Besides, this paper introduces a “file drawer” analysis according to Rosenthal [56] to estimate the severity of publication bias. The larger the coefficient, the greater the number of studies required to reverse this result, the more reliable the conclusions of the meta-analysis, and the smaller the relative impact of bias. After calculation, when *P*=0.05, Nfs = 10223, and *P*=0.01, Nfs = 7945, the fail-safe coefficient of this study indicate that the conclusion is more reliable.

This paper adopts Fail-safe, Egger's test (regression intercept method), and rank correlation test for further testing to test the publication deviation more accurately. The results are shown in Table 3. The fail-safe factor is *N* = 11495, indicating that if people want to overturn the TL effect, 11,495 documents are needed to get the opposite result. Egger's test results show that the *P* value is 0.88, which is not significant, and there is no publication bias. The level correlation test results, Tau values being −0.09 (*P*=0.58), suggest that there is no publication bias in the effect size.

### 4.2. Test of Heterogeneity

This study tests data for heterogeneity, which is a key step in synthesizing the global effect value from the practical value of a single study. The *Q* test results reflect the degree of heterogeneity of each effect size. If each effect size is heterogeneous, it indicates that the true error causes the difference of each effect size in the meta-analysis. Since the combination of variables can lead to sampling errors, the random-effects model should be applied. The test results are shown in Table 4. It can be learnt that *Q* (19) = 1713.0, *P* < 0.001, and *I*^2^ = 98.89%, indicating that the effect size of each study is heterogeneous. Among them, *I*^2^ greater than 75% means that the observed variation above 75% is caused by the true difference in effect size, reaching a high level of heterogeneity [56]. The values of Tau^2^ are 0.317, which means that 31.7% of the inter-study variation can be used to calculate the weight.

The heterogeneity test results show that the correlation between TL and project success is heterogeneous in the selected studies. Therefore, the random effect model is used in this study since it is more accurate for meta-analysis.

### 4.3. Theoretical Model and Test of Direct Relations

#### 4.3.1. Total Effect Size Test Result

According to the heterogeneity test results, the random-effects model was selected to test the main effects of the relationship between TL and project success (see Table 5). From the drawing, we can see that the overall test of the relationship between TL and project success, a total of 31 effect sizes (*N* = 6475), the overall correlation coefficient of TL and project success is 0.589 (*P* < 0.001), in 95% of the confidence interval is significant. When |*r*| ≤ 0.1, it is low correlation, 0.1 < |*r*| < 0.4 is medium correlation, and |*r*| ≥ 0.4 is high correlation. Based on this judgment, TL is positively correlated with project success. Therefore, hypothesis 1 is supported.

#### 4.3.2. Subdimension Effect Size Test Results

It can be seen from Table 6 that the *Q* test results of the heterogeneity of the relationship between each dimension of TL and project success are significant, indicating that each effect size is heterogeneous, and the random-effects model can be used. *N*'s loss of safety factor is more powerful than 500, showing no publication bias in each dimension's effect value.

From the dimensional meta-analysis results, the four dimensions of TL have some differences in their effect size; in detail, leadership charm is the largest (0.731) while intellectual stimulation is the most minor (0.619). According to Cohen's scale for social science research, correlations with values close to 0.2, 0.5, and 0.8 correspond to weak, moderate, and decisive effect sizes. Thus, leadership charisma reasonably correlates with project success, while vision motivation has a fragile relationship. As a result, hypothesis 2a–d is accepted.

#### 4.3.3. Moderation Analysis

As can be seen from the above, there is significant heterogeneity in the effect sizes for the meta-analysis in this paper. To further analyze the heterogeneity source, random-effects models are also adopted to test whether mediating variables, cultural background (Eastern culture, Western culture, and others), and literature publication types (journal papers, thesis).

The results in Table 7 show that whether to participate in the intermediary variables has a significant moderating effect on the relationship between TL and project success (*Q* = 336.669, *P* < 0.001). In the presence of intermediary variables, TL (*r* = 0.649, *P* < 0.001) and the correlation coefficients of project success were significantly higher than those of Western cultural background (*r* = 0.452, *P* < 0.001). Hence, hypothesis H3 is supported.

The cultural background also significantly moderates the relationship between TL and project success (*Q* = 55.641, *P* < 0.001). The empirical results indicate that TL in Eastern cultural backgrounds can play a more critical role in influencing project success. Thus, hypothesis H4 is supported.

Similarly, the literature publication has a significant moderating effect on the relationship between TL (*Q* = 214.251, *P* < 0.001) and project success. Under the dissertation type, the correlation coefficient between TL (*r* = 0.765, *P* < 0.001) and project success was significantly lower than that of the journal paper type (*r* = 0.513, *P* < 0.001). Therefore, it assumes that H5 is accepted.

## 5. Discussion and Implications

### 5.1. Discussion

This paper conducts an in-depth analysis of the empirical research on the relationship between TL and project success based on the meta-analysis method. It mainly focuses on the relationship between the various dimensions of TL and project success and the moderating role of the mediator variables, cultural background, and document type. Therefore, the following conclusions are drawn:

Firstly, the results suggest that TL can positively influence project success, in line with previous studies. The significant challenges of modern society and the increasingly different business environment require people to re-examine leadership research and change the traditional concepts and ways of thinking about leadership in the construction industry. A study by scholar Kissi [57] confirmed the necessity of project organizations to cultivate TL behavior to improve performance. By summarizing traditional team-building practices, Do [58] found that transformational leaders are more likely to enhance team members' understanding of project goals, roles, and responsibilities, interpersonal communication, and problem-solving skills, which will also help affect project success.

Secondly, this article's four dimensions of TL can improve project success in a cooperative-friendly way. To be specific, correlation strength is leadership charm, individualized consideration, idealized influence, and intellectual stimulation. Perhaps most empirical research on TL focuses on business operations, and the number of research samples in the construction context is relatively tiny. Stanislas [59] analyzed the indicators that affect sustainable construction and found that the personal charm of the project manager is one of the crucial indicators that can improve leadership effectiveness. Zia [60] reckoned that the emotional intelligence of project managers could improve partnerships and promote effective communication between project members. Maqbool [61] pointed out project managers with high emotional intelligence who bear the desired competencies and exhibit transformational leadership behavior are influential leaders and ensure higher success in projects than their counterparts. Also, Shafi [7] also indicated that idealized influence, intellectual stimulation, and inspirational motivation greatly influence organizational innovation. Many studies support this article's results [62, 63]. Therefore, the results of this article will help construction companies choose the right project manager for the project. At the same time, TL should pay attention to the rational use of the complementarity and dependence between various dimensions in the management process to promote project success.

Thirdly, mediating variables, cultural background, and document types are all sources of heterogeneity. Through a systematic review of meta-literature, this article finds one or more intermediary variables in most existing empirical models, such as knowledge learning, psychological capital, interorganizational relationships, and innovation atmosphere. Scholar Qaisar introduced psychological capital as an intermediary variable to construct a model and found that it negatively affected the relationship between the two. The existence of positive mediating variables will positively impact the relationship between project leadership style and performance, and vice versa. Under the East and the West's different cultural backgrounds, the influence of TL on project success is significantly different and regular. Under the environment of Eastern culture, the impact of TL on project success is higher than that of Western civilization. In particular, influenced by traditional Confucian culture [3, 64], high power distance, and collectivism, low-level project members in Chinese construction organizations are more likely to follow or accept organizational tasks assigned to leaders. However, the project members under a Western cultural background are more inclined to individualism, reflecting their ability and value [65]. Therefore, the construction project members under different cultural backgrounds will have other internalized explanations when facing the same leadership style, resulting in differences. Under the experience of Eastern culture, TL has a more noticeable impact on project members than in Western countries, resulting in a higher project success rate. In journal papers, more studies have been found to study the relationship between the two, and a large number of research scholars tend to establish empirical models to explore the boundaries of the two through different variables, which is also the direction of future research.

### 5.2. Theoretical Implications

On the one hand, this research enriches and extends the development of TL and project success theory. Through a meta-analysis, the reasons for the inconsistent conclusions on the relationship between TL and project success in past studies have been identified, and a focused comparison of the impact of different dimensions of TL and project success is conducted. The research results show that TL has a positive and significant relationship with project success, which provides a new research perspective for improving project success. TL and its impact on the success of the project have been reviewed in previous studies, mainly from the perspective of the overall impact of TL on the success of the project; this is far from enough. Therefore, this article analyzes and explains the differences in previous research results as a whole and helps to clarify the indistinguishability of the project success relationship caused by the mixed use of TL concepts. It can provide more accurate estimates of TL performance in different dimensions and dig deeper. The essence of TL's influence on project success is analyzed, and the impact of TL's dimensions on project success is sorted.

On the other hand, this article enriches and refines the boundary conditions and scope of application that influence the success of the TL project. Based on the empirical data analysis of the former National People's Congress, by further refining the moderating effects of the existence of mediating variables, document type, and cultural background, on the relationship between the two, a detailed discussion of the mechanism of TL and project success can be realized. The research results reveal the precise path of transformational leadership influencing project success, enriching and perfecting the existing project success model research. This article helps to understand TL-style project managers' internal laws of successful project operation and consolidates academic support for project management success in construction projects.

### 5.3. Practical Implications

This study provides several practical implications for construction companies and leaders. First of all, it helps construction companies preferentially select project managers. The results show that TL's leaders enhance team cohesion and mutual understanding, create a harmonious working atmosphere, promote the open exchange of ideas and analyses between project teams, and emphasize developing followers' self-management or self-leadership skills. In particular, selecting talents with strong leadership charm and abilities is more conducive to establishing a highly reliable organization for the project to cope with today's complex and changing international environment.

Then, the project managers should focus on their words and deeds on project members. Each project member can understand their mission and goal direction through vision incentives, translating into personal work goals. Inspiring leadership behavior through intelligence can create a challenging organizational atmosphere. This can make the project members more innovative and encourage them to express their ideas. The project manager actively cares about the organization's tasks and the needs of the project members, recognises the uniqueness and diversity of the beliefs and values of the project members, and provides corresponding support. Project managers should improve their own leadership charisma to enhance the self-confidence of members. At the same time, when making decisions, project leaders must have individualized considerations and seek more opinions from members to improve the identity and loyalty of project members. For example, in the Hong Kong-Zhuhai-Macao Bridge [66], well-trained professional subcontractors need better treatment, stable commitment, professional training, improved working conditions, genuine care, and on-site management for workers on-site. Therefore, it helps the Hong Kong-Zhuhai-Macao Bridge to achieve great success.

Finally, the construction project managers require to be trained in technical and soft leadership skills. The former ensures that project managers clearly understand and apply project management methods. The latter helps to adapt these methods to the specific social and cultural environment of the construction project. Thus, TL's leaders must make full use of the new generation of information technology, such as 5G, BIM, robots, etc. In the whole life cycle of project construction, they should lead the project members to achieve project success [67]. Also, they need to learn to use knowledge management and scenario deduction to make decisions, create a working environment that is most suitable for project members, and avoid limiting leaders' behaviors to a certain level. Meanwhile, as a survey concluded, different leadership styles are ideal for various projects [68]. So, it is necessary to adopt a diverse leadership style that adapts to the organizational environment to balance administrative tasks and meet the requirements of project members.

## 6. Limitation and Future Research Directions

There are several limitations that are worth mentioning. Firstly, the meta-analysis method only includes the analysis of the Pearson correlation coefficient when selecting samples, which will lead to the loss of some models. The removal of samples due to the inability to obtain effective effect sizes may affect the relationship in this article. Secondly, there is a limitation of potential moderating variable analysis. This study examines the potential moderating effects of situational features, design features, and measurement features, but different research samples will be affected by other factors. Future research can further explore other mediating factors, such as stakeholder relationships, psychological empowerment, individual values of project members, etc., to understand why certain construction activities can succeed while others fail.

## 7. Conclusions

There is a growing amount of research on the relationship between TL and project success, but the findings lack consensus. This meta-analysis provides more statistically valuable and accurate results for the general relationship between TL and project success by overcoming a single study's sampling error and sample size limitations. In addition, the moderating effects can be further tested to explore the influence of the existence of mediating variables, cultural background, and document types on the relationship of TL and project success and the inconsistent results of extant studies. In this way, a comprehensive theoretical framework is constructed for this study. The findings of this paper can provide better insights for choosing the right development strategy and improve leadership effectiveness to promote the project's sustainable development under the Industry 4. 0 era.

## Figures and Tables

**Figure 1:** The theoretical research model.

**Figure 2:** The flowchart of study selection.

**Figure 3:** Funnel plot of standard error by Fisher's *Z*.

**Table 1:** Definitions of project success.

Author	Definition
Edward [27]	Project success covers quality, time, cost.
Bryde and Robinson [28]	Project success includes pre-success, successful completion, and successful operation.
Kim and Reinschmidt [29]	The leading indicators of project success are customer satisfaction, quality, duration, cost, and other complex indicators.
Gabriella Cserháti [30]	There are five criteria for project success: efficiency, impact on a customer, impact on the team, business and immediate success, and preparation for the future.
Joslin and Müller [31]	Project success measurements include the iron triangle “time-cost-quality” and customer satisfaction.
Wang et al. [32]	Project success includes project efficiency, organizational benefits, project impact, stakeholder satisfaction, and future potential.
Luo et al. [33]	Project success includes time, cost, quality, health and safety, environmental performance, participants' satisfaction, user satisfaction, sustainability, and commercial value.

**Table 2:** Descriptive characteristics of the studies.

Author (time)	Category	Sample	Author (time)	Category	Sample
Odusami (2003)	(Y, J, W)	60	Xiang Ding (2017)	(Y, J, E)	162
Ralf Müller (2007)	(Y, J, W)	400	Yang Liu (2017)	(Y, T, E)	152
Arago'n-Correa (2007)	(Y, J, E)	408	Amin Akhavan (2017)	(N, J, W)	470
Anne Nederveen (2010)	(Y, J, E)	2	Yanchun Zhang (2018)	(Y, J, E)	251
Liu Xiaoyu (2011)	(N, J, E)	450	Jingting Shao (2018)	(Y, J, E)	79
Li-Ren Yang (2011)	(Y, J, E)	213	Lianying Zhang (2018)	(Y, J, E)	365
Kun-Shan Wu (2012)	(N, J, E)	106	Mustafa Raziq (2018)	(Y, J, W)	248
García-Morales (2012)	(Y, J, E)	168	Jae-Seung Hwang (2018)	(Y, J, E)	105
Susanne Braun (2012)	(Y, J, W)	360	Danting Li (2019)	(N, T, E)	201
Panagiotis Trivellas (2013)	(N, J, E)	97	Manandhar Sunitha (2019)	(N, J, E)	200
Huey-Wen Chou (2013)	(Y, J, W)	92	Floris (2019)	(Y, J, W)	37
John Kissi (2013)	(Y, J, E)	112	Li Danting (2019)	(N, T, E)	201
Muredeni Liphadzi (2015)	(N, J, E)	110	Doan (2020)	(N, T, W)	325
Assefa Aga (2016)	(Y, J, W)	224	Hassan Shah (2020)	(Y, T, E)	150
Zhang Lian-Ying (2016)	(N, J, E)	237	Jabran Khan (2020)	(N, J, W)	256
Aga (2016)	(Y, J, E)	200			

*Note*. Y: the existence of mediating variables; N: the absence of mediating variables; W: Western culture; W: Eastern culture; J: journal; T: thesis.

**Table 3:** Publication bias test.

Leadership style	NFS	Egger's test	Tau	Trim and fill		
				Observations	Adjusted value	Change value
TL	11495	1.01 (*P*=0.88)	0.09 (*P*=0.58)	0.589	0.301	0.288

**Table 4:** Results of the heterogeneity test.

Leadership style	*N*	Heterogeneity test				Tau^2^				
		*Q*	Df (*Q*)	*P*	*I* ^2^		Tau^2^	SE	Variance	Tau
Transformational leadership	31	1713	19	<0.001	98.891		0.317	0.132	<0.05	0.563

**Table 5:** Total effect size element analysis results as the test.

Leadership style	Model	*K*	*N*	95% CI			*Z*	*P*
				Point estimate	Lower	Upper		
TL	Random	31	6475	0.589	0.398	0.732	5.187	<0.001

*Note. K* = number of studies; *N* = sample size; *r* = effect size; 95% CI = confidence interval around *r*.

**Table 6:** Dimensional meta-analysis results.

H	Heterogeneity test			*K*	*N*	95% CI			Two-tailed test		NFS
	*Q*	df	*P*			Point estimate	Lower	Upper	*Z*	*P*	
H2a	1589.59	10	<0.001	20	3243	0.731	0.612	0.817	8.366	<0.001	6376
H2b	824.79	10	<0.001	12	2948	0. 673	0.487	0.811	5.638	<0.001	5178
H2c	484.94	8	<0.001	8	2149	0.619	0.482	0.785	5.842	<0.001	3154
H2d	1093.4	9	<0.001	10	2543	0.721	0.576	0. 822	7.051	<0.001	6602

*Note. K* = number of studies; *N* = sample size; *r* = effect size; and 95% CI = confidence interval around *r*.

**Table 7:** Results of moderation analysis.

Moderating variable	Leadership style	Heterogeneity test			Sort	*K*	*N*	95% CI			Two-tailed test	
		*Q*	df	*P*				Point estimate	Lower	Upper	*Z*	*P*
Mediating variable	Transformational leadership	336.669	2	<0.001	Y	23	1254	0.573	0.622	0.817	8.546	<0.001
					N	8	1583	0.469	0.608	0.795	7.128	<0.001

Cultural background	Transformational leadership	55.641	2	<0.001	E	10	2319	0. 893	0.587	0.831	5.748	<0.001
					W	17	1826	0.759	0.452	0.776	5.682	<0.001
					O	4	1382	0.723	0.632	0.797	8.426	<0.001

Document type	Transformational leadership	214.251	2	<0.001	J	3	781	0. 611	0.467	0.834	5.678	<0.001
					T	28	2825	0.677	0.512	0.792	5.7843	<0.001

*Note.* Y: the existence of mediating variables; N: the absence of mediating variables; W: Western culture; E: Eastern culture; O: other; J: journal; T: thesis; *K* = number of studies; *N* = sample size; *r* = effect size; 95% CI = confidence interval around *r*.

## Data Availability

The data used to support the findings of this study are available from the corresponding author upon request.
